# College English Teaching Platform Optimization under Cross-Media and Mobile Internet Environment

**DOI:** 10.1155/2022/9672463

**Published:** 2022-05-11

**Authors:** Wei Wang

**Affiliations:** Quzhou University, Quzhou 324000, China

## Abstract

In the construction of a new teaching model and digital learning environment suitable for the development of The Times, cross-media and mobile Internet environment teaching is playing an increasingly important supporting role. Educational software is one of the most widely used educational software in the world today. More and more colleges and universities are using platforms to assist English teaching and exploring effective ways to promote English teaching reforms by using the cross-media and mobile Internet environment, so as to improve the students' course learning effect. Based on the characteristics of college English majors, this paper discusses how to use the platform to assist English teaching. The cross-media and mobile Internet application environment university teaching optimization platform is a good resource sharing, communication, cooperation, and learning space, as long as teachers of innovative ideas and the localization of the platform, the practical application, and the individuality can give full play to the advantage of the platform and practice the traditional teaching method and modern media and mobile Internet environment information technology complement each other, promoting the improvement of English teaching effect. The aim of this study is to construct the college English teaching system optimization model, emphasizing that students are the most important ecological factors in this model, and that teachers, teaching elements, information technology, environment and other factors play a role in the appropriate ecological niche and change synergistically. The whole system of college English teaching is in a dynamic balance through the circulation and exchange of material, energy, and information among the factors inside and outside the system. Starting from the external environment of mobile Internet, the teaching method of professional basic mathematics course is deeply deconstructed, and the teaching design idea based on the teaching content is the main teaching line, and the teaching interaction of students' immediate feedback is the secondary teaching line that is proposed. The college English curriculum reform practice is carried out in combination with mobile applications. In specific teaching practice, smart classroom design is taken as the theoretical carrier, auxiliary platform is applied to realize teaching feedback interaction, and the teaching concept of mixed learning and collaborative learning is realized with a real-time feedback teaching interactive tool.

## 1. Introduction

College English teaching is a systematic project, which requires students to have the ability of comprehensive language application. Listening, speaking, reading, writing, and translation are five core parts. In order to achieve this teaching goal, the research and teaching staff in the Chinese universities have carried out various research studies and practices on how to improve the students' English application ability, but the results have not reached the expected goal. With the continuous development of Internet technology, multimedia teaching has been widely introduced into the classroom of colleges and universities [1], which has brought a great impact on traditional English teaching. Multimedia teaching is easier to be accepted by students.

Clearly put forward, the school should make full use of modern information technology, based on the Internet media and mobile Internet application of optimization of the teaching platform and environment university classroom English teaching mode, use of network technology, enrich teaching forms, and change the traditional classroom [2], in order to meet the demand of students autonomous learning and individualized learning direction. The construction of college English teaching model and college application teaching optimization platform based on corpus and cross-media and mobile Internet environment comes into being under the background of allowing students to learn English anytime and anywhere without time and place restrictions through the Internet.

With the advent of the information society, people are increasingly using computers and networks. Information technology has penetrated into every field of people's life, and education is no exception. Information technology has greatly promoted the reform of educational means, mode, system, concept, and so on and made many ideas of teaching reforms better realized. In 2 of higher school teaching quality and teaching reform projects in [3, 4], the Ministry of Education intend to by means of information technology deepen the reform of teaching and talent training mode reform, as the top of the 12 projects, and clearly put forward the construction of 1500 fine courses and will the lesson plans on the Internet, promote quality education resource sharing [5]. In terms of foreign language teaching, the requirements of college English course teaching [6] and college English course teaching [7] both clearly put forward that “We should make full use of the opportunities brought by the development of multimedia and network technology, adopt new teaching mode to improve the original single classroom teaching mode based on teachers' teaching;” The new teaching mode should be supported by modern information technology, especially network technology, so that English teaching will develop toward personalized learning, learning without time and place restrictions, and active learning. The cross-media and mobile Internet environment university applied teaching optimization platform is an indispensable environmental foundation to promote the rapid development of teaching informatization and plays an important supporting role in the construction of a new teaching model and digital learning environment suitable for the development of The Times [8]. Most colleges and universities have purchased, developed, and constructed the university application teaching optimization platform of cross-media and mobile Internet environment. As one of the most widely used educational software in the world [9], educational software has been selected by many well-known universities and international top business schools to strengthen network teaching and assist classroom teaching in colleges and universities [10]. At present, the cross-media and mobile Internet environment university application teaching optimization platform has been widely used in the world, and gradually promoted in domestic universities [11]. More and more colleges and universities are using the cross-media and mobile Internet environment college application teaching optimization platform to assist English teaching, exploring effective ways to use the Internet to promote English teaching reforms, so as to improve the students' course learning effect.

At present, college English teaching in most higher vocational colleges is still based on the teacher-centered teaching mode. The student is to basically listen to the teacher in class where personal interpretation of the text content is given priority to; through typical text content learning English grammar, words, etc., is the main reading comprehension on after-school exercises, which completely ignored the students' reading, writing, listening, speaking, and other various aspects of ability training; in this mode, the students in order to pass the national college English Test Band four and six as the goal. College English is test-oriented English, which makes a large number of “mute English,” as unable to carry out normal communication through English. Some colleges and universities have seen the disadvantages of this model and have begun to make comprehensive changes in English teaching to improve students' English application ability [12, 13]. Observing the English teaching goal, the main aspect can be divided into several levels, in which the means through the national level English test is predominant; at present, most of the courses in English for the purpose of higher vocational colleges are still a subject to a student through the national English level test in the English level as the goal; students are required to improve by learning English. Students can learn about foreign language works of their major through English. Through the development of basic English courses, on the one hand, students' English reading, writing, and communication abilities can be further improved [14]. On the other hand, “passing grade” is taken as an important standard to measure the students' English level. Second is the combination of English courses and featured majors cultivates talents with a certain professional English ability. The college English teaching method mainly focuses on strengthening the students' English communication ability, while taking other aspects into account. The main teaching method is to improve the students' English application ability through communication with foreign teachers [15]. Third is through the English teaching reform, according to different characteristics of students, through the combination of information technology and college English teaching, which carries out targeted teaching, to train various kinds of applied professional and technical personnel, improve the students' English application ability, promote students to use English in their professional level, to cultivate students in listening, speaking, reading, writing, and other various aspects of ability. Through continuous summaries in practical teaching, scholars put forward the classroom introduction method of college English, taking the cultivation of students' literacy as the starting point, and focusing on the cultivation of computational thinking in college English teaching [16]. As the education model transformation trend of computer science and technology major teaching form has been updated; in literature [17], this paper discusses the lesson “for” the new curriculum provides the high quality resources, improves the classroom efficiency of positive influence, puts forward the micro class with the form of “application of teaching” change teacher's role, advocates independent learning strategies, and optimizes the cultivation of college English compound talents. According to the teaching difficulties of college English graduate courses in teaching practice, literature [18] organically integrates college-applied teaching and traditional teaching mode and constructs a mixed teaching mode from four aspects: teachers' in-class teaching, teachers' after-class support, students' self-learning after class, and college-applied teaching. Literature [19] stimulates the students' learning potential and subjectivity by “flipping” the traditional teaching mode and making use of its features such as short and concise videos, clear teaching information, reconstructed learning process, and convenient review form. Based on the discussion of college-applied teaching and the teaching situation of college English in China, this paper aims to improve the students' practical application ability and innovation ability by applying college-applied teaching. Literature [20] proposed that the reverse teaching method of scientific research cases should be introduced into college English teaching, and teaching cases should be designed from the perspective of improving various abilities of professional training. In view of the new engineering education, literature [21] proposed the college English teaching reform oriented to the cultivation of applied practical ability, and explored the teaching methods of college English from the design of teaching content and teaching mode. Literature [22] deeply studied the teaching design model of a microcourse teaching mode in college English courses in higher education and discussed the theoretical feasibility through practical MOOC environment practice. Literature [23] re-examines the course positioning of college English, analyzes the correlation between college English course content, big data, and artificial intelligence, and puts forward targeted teaching reform measures to further increase the teaching emphasis of this course under the background of artificial intelligence.

The optimization of college English classroom teaching is a hot issue in the reform of college English teaching, which is directly related to the success of the reform. Scientific and effective personalized learning methods and teaching methods under the network environment are the important content of the optimization of college English classroom teaching, and the fundamental guarantee for improving the quality and effect of college English teaching and improving the actual effect of college English teaching in China. Under the background of college English teaching reform carried out by the Ministry of Education, the research of this topic is based on the practice of teaching reform, to explore the optimization framework of college English classroom teaching in the network environment and to emphasize the construction of independent learning strategies and the concept of teacher development in the network environment. The research results are of practical value and practical significance for building the ecological balance of informationized foreign language teaching and improving the effectiveness of college English teaching reforms.

## 2. Analysis on the Relationship between Cross-Media, Mobile Internet Environment, and College English Teaching Optimization Platform

### 2.1. College English Course Teaching Method in a Mobile Internet Environment

The innovation of the research lies in that the instant delivery and feedback of teaching knowledge information are considered in the research. The interactive teaching tool of instant feedback of mobile terminals is explored as the software platform, and the students' mobile phones are used as the hardware teaching auxiliary environment. In the learning process, the initiative and enthusiasm of students are brought into play by the means of mobile Internet technology. The main idea of the research is to take the teaching content as the main line of teaching, the interaction of students' immediate feedback as the secondary line of teaching, combined with a mobile phone application to carry out the basic mathematics curriculum reform practice of the computer major. We aim to achieve a comprehensive application of cooperative learning and mixed learning to explore the teaching reform of basic mathematics courses for computer majors. In this study, the main body of students is mobilized through the application of instant feedback teaching interactive tools (Blue Ink Class App and Learning Pass App). The specific framework is shown in Figure 1.

According to the research framework of the subject, the teaching method under the mobile Internet environment is mainly explored. The specific research method is to use the auxiliary platform to realize the teaching feedback interaction and use the instant feedback teaching interactive tool to realize the teaching concept of mixed learning and collaborative learning.

The concept of blended learning is mainly an organic combination of face-to-face classroom learning and online learning. Different information technologies are applied in the form of technology and combined with teaching methods to achieve the optimal learning effect. In this study, the real-time feedback teaching interactive tool of mobile Internet is used as an auxiliary platform for university application teaching optimization in the cross-media and mobile Internet environment, and the optimal teaching effect is achieved by the real-time interactive feedback. Specific combination of blue ink class APP is as follows:

1. Using the “resources” in the application, teachers guide students to learn microlesson resources and stone teaching materials and share them with students other network resources. Online learning resources can be published in the auxiliary platform to facilitate students' independent learning.
2. Use “Q&A discussion(question/answer discussion)” in the application to collect students' questions in class and mobilize students' enthusiasm to participate in course learning by mobile means.
3. Use the “test” in the application to conduct in-class tests, so that teachers can master students' understanding of knowledge points in the first time.
4. Use the “brainstorming” in the application to mobilize students to have interactive discussion in class, including online discussion or private letter questions (teachers answer them individually), so as to avoid the situation that students are unwilling to ask questions face to face.

The concept of collaborative learning is to organize students in a group and enhance their professional knowledge through mutual assistance. The pre-class preview and classroom participation of college-applied teaching rely on the communication between student groups and team members to internalize knowledge into the heart. Collaborative learning can eliminate students' helplessness in network learning, experience different roles and accept different views in the discussion, and achieve the goal of collaborative knowledge construction. Teachers provide clear learning tasks, organize students to actively participate in cooperative learning and teaching activities, and make invisible knowledge apparent in communication and interpretation.

College English teaching corpus across media and carrier of the mobile Internet environment university-applied teaching optimization platform is the campus network based on Internet technology, through independent development software and using mature software, which is set up across the media and mobile Internet application environment university teaching optimization platform-dedicated server, building a service of college English teaching corpus of the network platform. The main steps are as follows: collation and collection of college English teaching corpus, development, and installation of software. In corpus construction, the collection of advanced technology is done at home and abroad. The basic English curriculum system is based on English language knowledge and application skills, learning strategies and cross-cultural communication, and integrates various teaching modes and means. The basic English curriculum of this teaching reform is shown in Table 1.

Students are actively encouraged to log in to the campus network student cross-media and mobile Internet environment University application cross-media and mobile Internet environment university application teaching optimization platform, using online classrooms for teaching guidance, each student must study online for no less than 80 hours in a semester. Teachers should conduct real-time regulation and guidance on course learning in the management modules of the platform, such as “Course Center,” “Operation System,” “Online Q&A,” “Student files,” “Discussion and Exchange,” “Resource Center,” etc. Teachers should upload courseware in class to the center of multimedia courseware for the students to download, actively encourage students through the platform of “study BBS” columns and teachers to learn the content of text, the teacher should answer questions quickly, provide students with online answers or suggestions for the curriculum, teaching methods, etc., guide students through the platform of “online learning” in the “extension of knowledge” to study, to provide rich learning resources for students, let students appreciate the foreign original films and documentaries, improve students' interest in learning English, promote mutual learning among students, and encourage students through the platform between “online communication” function to use English to communicate, to improve students' ability to use English in practice.

### 2.2. College English Cross-Media and Mobile Internet Environment Teaching Optimization Platform Optimization

Across different media and mobile Internet environment at the university of application and mobile Internet media environment university-applied teaching optimization platform across media and mobile Internet application environment university teaching optimization platform “has strong core functions, make teachers can effective management courses, content, making operation, and strengthening cooperation, to help schools achieve related to teaching, communication, and evaluation of important goals.”

Virtual classroom is a collaboration tool of the college application teaching optimization platform system for transmedia and mobile Internet environment. It enables teachers and students to participate in real-time courses and discussions and view records of previous collaborative sessions. Teachers can use system controls to manage conversations, control access to and interact with other participants in the conversation, and use whiteboards to view content, web pages, and drawings. Chat is a part of the virtual classroom but can also be accessed individually. It allows users to turn on only the “chat” feature of the virtual classroom. Collaboration tools can be used to host live online class discussions, sessions, and physical and public time type Q&A forums. Guest lecturers and subject matter experts can also use collaboration tools to talk with the class, and the college application teaching optimization platform system has powerful assessment and evaluation functions. Through the test manager, teachers can create and organize tests, exams, and surveys and can get instant test results' feedback; through the question bank manager, teachers can establish their own test bank and can repeatedly generate random test papers from the test bank. The test can move after the completion of the teacher to student's answer for grading and evaluation, through an online grade book to publish and test all the student achievement. The online grade book can be generated by a user or by a breakdown test score report, and a spreadsheet view function is a powerful tool for management course grade, you can add record book breakdown, input results, set the grade weighted, rank your grades and divide your grades. The structure diagram of the platform teaching process is shown in Figure 2.

The course construction framework teaching process structure diagram of university application teaching optimization platform is built based on the university application teaching optimization platform of cross-media and mobile Internet environment, and the course portal is formed according to the requirements of course construction. The course tasks are distributed according to different class progress. Taking the content of paradigm in propositional logic as an example, the specific tasks are three task points, the concept and solution of conjunctive paradigm and disjunctive paradigm, minor term and major term, and the steps of main disjunctive (conjunctive) paradigm of the propositional formula.

### 2.3. Specific Application of the College English Teaching Optimization Platform in the Context of Cross-Media and Mobile Internet

1. Make teaching plans and lay a solid teaching foundation by using the university application teaching optimization platform in the cross-media and mobile Internet environment.
2. In the first semester after freshman's admission, teachers should formulate English teaching tasks through the university application teaching optimization platform of cross-media and mobile Internet environment, make relevant multimedia courseware, and carry out teaching tasks according to the teaching time and place assigned to teachers by the platform. Through the plan, teachers can prepare for teaching in advance and communicate with students in time. Students can also learn actively by understanding the teaching plan.
3. Through the use of network classroom, teachers guide students to combine “teaching and learning”
4. Through explaining students the use of college application teaching optimization platform in campus cross-media and mobile Internet environment, students are required to prepare before, during, and after class and take the network platform as a bridge to continuously study independently, so as to improve the teaching effect. This paper focuses on the comprehensive basic courses of college English, namely, “audio-visual speaking” and “reading, writing, and translation.” The required courses of college English in the three universities are shown in Table 2.
5. A: in colleges and universities under the guidance of the school teaching target, according to the three stages of teaching characteristics, the school curriculum is divided into two parts: the basic phase and improve the phase of the curriculum are mainly comprehensive basic course and application courses, comprehensive foundation courses as required courses, including the following two classes: “audio-visual” and “writing and translating.” The courses in the improvement stage are required courses, general courses, or elective courses, depending on different levels, which are divided into four categories, as shown in Table 3.
6. The platform application enables teachers and students to interact with each other and stimulates students' interest in learning
7. Students communicate in English through the network platform and carry out practical exercises by setting up situations. Linguists study showed that any kind of language, an effective way to rapidly increase, is formed in the surrounding to communicate in the language environment, so the teacher must use the network platform to set up a situation as much as possible on the knowledge, let the students practice in the situation, said through the exchange between students, making students learn music not only can improve the efficiency of classroom teaching but can also promote students' interest in English. As shown in Figure 3 (college English class/audio-visual teaching evaluation chart).

### 2.4. Experimental Design

As mentioned above, college English teaching in most universities also contains the potential pressure of CET-4 (College English Test Band 4), so it is inevitable to involve CET-4 and CET-6 in the teaching content, especially CET-4. According to the survey, most teachers spend more or less time in class to train students before CET-4. As shown in Table 4, only 11% of teachers never teach anything related to CET-4. On the other hand, the students' learning motivation is largely due to external factors test (level 4) drive, some students believe that get a certificate iv can help them get a better job, or get a university diploma and degree certificate (C) school students, so students also take a large part of time in class for learning and the levels four/six of tests.

The new teaching mode requires student-centered and teacher-led teaching. This role of teachers and students has different manifestations in different situations. For example, teachers may be trainers or organizers. Students may be receivers of information, collaborators, and so on. Obviously, the roles of teachers and students in college English teaching are characterized by diversification. See Table 5.

## 3. Results and Analysis

By using information technology to establish a university teaching optimization platform for campus cross media and mobile Internet application environment, the university has not only comprehensively changed teachers' classroom teaching methods but also guided students to use them and cultivated students to form a good habit of self-study. Students have changed from passive teaching to active teaching. While optimizing the teaching platform through cross media and mobile Internet environment, they have also changed their learning methods and improved their interest in learning English. The attendance rate in English class has increased, and the attendance effect is shown in Figure 4.

In terms of the improvement of English scores, 32.29% of the students said that their English scores had been greatly improved, 44.42% said that they had improved, and only 12.42% came to the conclusion that there was no change. 69.37% of the students choose listening comprehension and translation as the most obvious aspects to improve their English through new teaching mode. In the original teaching mode, the biggest difference is the aspect: 36.3% of the students proposed to increase the application of network teaching, pay attention to cultivate students' independent learning ability, 31.8% of the students chose to improve students' English comprehensive quality, enhance students' communication ability. Together, nearly, 80% of the students believe that the teaching reform, on the one hand, has changed the original teaching mode, and on the other hand, it has enhanced the ability of students to study independently and cultivated the good habit of students' independent learning. In terms of improvement in teaching, 56.36% of students think that the current teaching progress is fast, while students' own learning is poor, and they hope teachers to adopt differentiated teaching, as shown in Figure 5.

See from Figure 5, the author thinks that based on cross-media and mobile Internet environment at the university of application, optimize teaching platform can obviously change the English teaching mode, improve the quality of teaching, students can also through the network autonomous learning platform for autonomous learning, to improve students' English comprehensive ability, especially speaking and listening to improve evident, however, Since the platform is still in its initial stage, it needs continuous improvement. Meanwhile, the purpose of teaching students according to their aptitude has not been fully reflected. In the future, differentiated teaching for students will be further enhanced.

Students' English scores can also reflect the change in teaching mode and bring practical changes to students. By checking the English scores of students in the same class in the academic administration system, it was found that the average score increased from 68.8 to 70.8, and the number of students who reached the qualified line increased from 72 to 128, and the number of students with more than 85 points increased from 24 to 35. By checking the attendance records of students in English classes, it was found that the attendance rate increased from 80% at the beginning of the semester to 96% at the end of the semester, as shown in Table 6.

The above data fully reflect that the university has combined information technology with teaching, established a university teaching optimization platform for cross media and mobile Internet application environment, guided students' autonomous learning, improved teaching quality, and improved students' ability to use English.

The results show that the content of online learning is “multitasking,” of which the top two and more than half are listening practice and writing practice. This result is consistent with the statistical results of the first and second questions, and also related to the nature of college English courses. College English courses “focus on English language knowledge and application skills, cross-cultural communication and learning strategies,” while college English courses are “both instrumental and humanistic.” It can be seen that the cultivation of language skills is one of the main tasks of college English courses. The content of online learning also depends on the capabilities of the platform used, as shown in Figure 6.

In terms of teaching behavior in the cross-media and mobile Internet environment, the scores of teachers in ordinary universities were significantly higher than those in 211 universities. Compared with the total score of effective teaching behavior, the scores of teachers in 985 colleges and universities were significantly higher than those in 211 colleges and universities, and those in ordinary colleges and universities were significantly higher than those in 211 colleges and universities.  Figure 7 can be more intuitive to see the comparison of scores of teachers in universities at the three levels in each factor. Each factor has a different weight,such as personalized teaching, multiple evaluation, face to face online, teacher support, and online learning.

In the third place were online jobs or tests. The biggest characteristic of this kind of platform is that the system automatically scores, so that teachers are liberated from the heavy homework correcting work. For example, a college involved in the survey uses the platform to require students to complete 10 sets of CET-4 simulation questions (excluding the composition) every semester. After students submit the questions, the system will give the scores of each question and the correct answers immediately. Many college English teachers also choose to use online platforms such as “jiaogai.com” and “Juku.com” to correct their compositions. See Figure 8.

In conclusion, learners' emotional experience plays an important role in studying the influence of cross-media multitasking on learning. Emotions are not only the influencing factor but also the result. This study inspires us to continue to explore the influence of cross-media multitasking on more emotions in the future research. Meanwhile, other aspects of learning, such as learning results and learning efficiency, should be considered comprehensively in the research, so as to discover more research results and improve the cross-media multitasking research.

## 4. Conclusion

Based on the literature analysis on cross-media multitasking, this study found that there is still a gap in the study on the impact of on-task cross-media multitasking on learning at home and abroad. Therefore, it can be applied for the future of the university teaching course designers and a line of teachers teaching model to provide necessary reference. According to the can depend on the results of the paper can also provide the necessary information for front-line teachers, make it realize the application of teaching shortcomings and the insufficiency, and puts forward some constructive solutions, For the future classroom teaching design and adjustment to do a good job in the corresponding preparation, to avoid the possible problems in the university-applied teaching. The next step is to establish a corpus for college English teaching platform of cross-media and mobile Internet, so that students can choose to learn according to their own needs and teachers can move.

## Figures and Tables

**Figure 1:** Research framework of the mobile Internet environment.

**Figure 2:** Teaching process structure diagram of university application teaching optimization platform based on the cross-media and mobile Internet environment.

**Figure 3:** College English reading and writing/audio-visual teaching evaluation chart.

**Figure 4:** English basic attendance rate in the first semester.

**Figure 5:** Data chart of 2013 and 2014 college English test scores of experimental class of English teaching reform in School A.

**Figure 6:** Online learning content.

**Figure 7:** Comparison of effective teaching behaviors of College English teachers at different levels.

**Figure 8:** Types of online learning platforms.

**Table 1:** Curriculum of the college English teaching reform.

Semester	Textbook	Grade	Score	Class
1	College English (1)	Basic English	6	16
2	College English (1)	Basic English	8	16
3	College English (1)	Basic English	8	12
4	College English (1)	Basic English	8	12
5	English courses of your choice	Improve English	4	8

**Table 2:** Compulsory courses of college English in three universities.

Colleges and universities A				Colleges and universities B		Colleges and universities C			
Autonomous learning		Reading and writing class	Audio-visual speaking lesson	Audio-visual presentation (self-study is arranged in this class)	Intensive reading class	Reading, writing and translation	Network video	Spoken language	Autonomous learning
Read and write	Listening	4 hours	4 hours	3 hours	2 hours	2 hours	3 hours	2 hours	Reading/writing/audio-visual/speaking
3 hours	3 hours								4 hours

**Table 3:** Specific pattern of course setting.

Phase	Foundation stage and improvement stage	The follow-up (specialization) stage
General requirements (level 1 starting point)	(1) Comprehensive foundation courses (1st to 4th semesters) (2) Advanced courses (general or elective courses after the fourth semester)	Professional English (compulsory courses, optional courses, bilingual teaching)
Higher requirements (level 2 starting point)	(1) Comprehensive foundation courses (1st to 4th semesters) (2) Advanced courses (general or elective courses after the fourth semester)	
Higher requirements (level 3 starting point)	(1) Comprehensive foundation courses (1st to 4th semesters) (2) Advanced courses (general or elective courses after the fourth semester)	
Note	This stage of the course is undertaken by the big external	This stage of the course will be undertaken by professional teachers from the university or each school

**Table 4:** Proportion of college English teachers teaching CET-4-related content in class.

	Always	Often	Sometimes	Once in a while	Never
Number	12	12	12	11	5
Percentage	23%	23%	23%	21%	10%

**Table 5:** Teachers and students on the role of teachers.

Teacher's role		Evaluators (%)	Trainers (%)	Organizers (%)	Assist (%)	Design and developer (%)	Guide (%)	Communicator (%)	Data organizer (%)
Teacher questionnaire	You think the teacher's role should be	32	38	68	61	58	58	53	41
	Your role in the actual teaching is	65	32	59	46	42	52	72	42
Student questionnaire	You think the teacher's role should be	50	71	51	64	41	58	64	46
	Your role in the actual teaching is	82	36	58	68	43	57	75	47

**Table 6:** Pass rate of College English Rank Examination for the experimental class of teaching reform of A university.

Name of the test	Registration number	Number of real test	By the number	Pass rate (%)
December 2013 English level test	38	33	14	40.82
June, 2014 English level test	91	86	46	51.75
December 2014 English level test	96	92	55	60.41

## Data Availability

The data used to support the findings of this study are available from the corresponding author upon request.

## References

[1] Deng F. (2020). The optimization research on college English classroom teaching under the network environment—based on the feedback report of college English stratified teaching in SASU. *Teaching English in China and America*.

[2] Wei Q. (2016). Research on college English teaching model optimization under information technology background: taking xi’an university as empirical analysis example. *International Technology Management*.

[3] Cai W. Q., Zhang Y. L. (2017). The optimization of college English teaching environment. *Journal of Jiamusi Vocational Institute*.

[4] Tian Z. (2020). Research on optimization of college English classroom teaching based on computer network environment. *Journal of Physics: Conference Series*.

[5] Yi H. E. (2015). Research and building of optimization measures of college English teaching. *International Technology Management*.

[6] Wang L. (2017). Study on the optimization application of computer assisted instruction in college art teaching. *Revista de la Facultad de Ingenieria*.

[7] Gupta A., Capponi A., Smith J. C. (2016). Optimization challenges in complex, networked and risky systems. *Research and Teaching Opportunities in Project Management*.

[8] Guo X. (2017). Construction analysis of ecological college English teaching model in computer network environment. *Journal of Computational and Theoretical Nanoscience*.

[9] Israel-Fishelson R., Hershkovitz A., Eguíluz A., Garaizar P. M. (2021). A log-based analysis of the associations between creativity and computational thinking. *Journal of Educational Computing Research*.

[10] Whitehouse H. (2015). Cross-sectorial relationships for education for sustainability. *CSR, Sustainability, Ethics & Governance*.

[11] Bo L. I., University B. N. (2016). Research on optimization of college Chinese teaching under the network environment. *The Guide of Science & Education*.

[12] Yan-Fei D. U. (2017). Exploration of college English teaching model in mobile Internet time. *DEStech Transactions on Environment Energy and Earth Science*.

[13] Feng L. I. (2015). The optimization of college English teaching mode in the independent college——college English graded teaching. *Theory Research*.

[14] Chen W. (2019). Optimization management and effective learning in SPOC blended learning applied in college English teaching. *Journal of Heilongjiang University of Technology (Comprehensive Edition)*.

[15] Sheng F. (2016). Research on the optimization of participatory teaching approach under the mode of subjective education:A case study on the lesson “anti-Japanese war”. *The Science Education Article Collects*.

[16] Cheng L. I. (2017). Under the network environment of university teaching computer optimization path to explore. *Education Teaching Forum*.

[17] Jing H. U. (2015). Study on mobile learning in college English flipped classroom teaching model. *Research on Higher Education of Nationalities*.

[18] Yan L. (2018). Optimization of mental health education methods for college students in new media environment. *Journal of Jiamusi Vocational Institute*.

[19] Jingting X. U., Liu H. (2019). Research on the teaching strategy optimization of architectural English course under the double orientation of EAP+EOP. *The Guide of Science & Education*.

[20] Chen Z. L., Liang X. T., Marxism A. O. (2018). Research on optimization of ideological and political education environment for college students. *Teaching of Forestry Region*.

[21] Bingyan H. E., Qun L. I. (2017). On the tendency of the internet-assisted teaching platform of moodle:as exemplified in English reading and writing of SISU. *Foreign Language and Literature*.

[22] Song L., Guo Y., Bai C. (2016). On the optimization of teaching in multi-levels of college mathematics under the system of credits. *Journal of Henan Institute of Science and Technology*.

[23] Hao L. V., Guo G. H. (2020). Optimization and design of teaching sections in college teaching competition—taking college physics for example. *DEStech Transactions on Social Science Education and Human Science*.

